The article "First-Aid System for Marathon Athletes Based on Telemedicine Technology" was published in 2022. Journal: Appl Bionics Biomech.

# First-Aid System for Marathon Athletes Based on Telemedicine Technology

**DOI:** 10.1155/2022/3335225

**Published:** 2022-09-06

**Authors:** Caixia Chen, Shuai Liu

**Affiliations:** ^1^The Faculty of Physical Education, China West Normal University, Nanchong, 637002 Sichuan, China; ^2^Physical Culture Institute, Hunan University of Humanities, Science and Technology, Loudi, 417000 Hunan, China

## Abstract

With the emphasis on sports in the region and the improvement of people's living standards, more and more people participate in various sports and activities including marathon, so that more and more cities are hosting or even vying for it. With the marathon, not only the joy of successfully holding the event, but also the pain of the contestants and even the sadness of sudden death. In order to reduce the occurrence of such problems, this paper studies the emergency system of marathon runners based on telemedicine technology. The experimental results show that the research on first-aid bears for athletes based on telemedicine technology can save a lot of time and managers, improve the efficiency of first aid by 3.45%, and provide first-aid services for injured athletes at the first time, so as to ensure the health of athletes, ensuring the confidence and well-being of athletes participating in the marathon.

## 1. Introduction

The marathon has become the most popular large-scale outdoor activity in recent years, but since it is an activity, there will always be some problems that may cause injuries to athletes. Failure to provide first aid to athletes after an injury could have serious consequences that no one can bear. However, the marathon is an outdoor activity, and it is difficult to provide face-to-face services. In addition, the current research results of the first-aid system for athletes are very scarce. Therefore, the research on the first-aid system for marathon athletes based on telemedicine technology has become the top priority.

No matter what arena, first aid for athletes is an important part of event protection. It can not only escort athletes chasing their dreams, but also a reflection of their ability to run competitions. The team has all done research on this. As part of a comprehensive campus health care system, Bartz-Smith sees injury care clinics as a cost-effective way to utilize a collaborative health care model to optimize patient care processes in the face of physician shortages [1]. Elkington and Hughes aim to ensure that when dealing with concussions in sports, the focus is on the safety and welfare of participants [2]. Since hamstring tendon grafts, despite being the first choice for knee ligament reconstruction, may not be of sufficient size, Oliveira et al. found the peroneus longus tendon as a new graft replacement [3]. Based on binocular stereo vision measurement and wireless sensing theory, Li and Zhang studied the measurement and analysis methods of athletes' motion displacement parameters, the main purpose of which is to explore the relationship between motion biomechanical parameters [4]. To better coordinate the management of athlete data collection, Nugraha created an information system to assist in the collection of athlete data [5]. Since the current system is not athlete-centric, Lombard proposed the idea that an understanding of their best practices needs to be established when considering high school athletes [6]. On the basis of literature research, Vysochina and Vorobioda made a systematic and generalized understanding of the psychological correction methods of athletes' personality in the modern Olympic movement [7]. It can be seen that the research on first aid for athletes has been very rich, but few people have put first aid for athletes on the marathon arena.

The article "First-Aid System for Marathon Athletes Based on Telemedicine Technology" was published in 2022. Journal: Appl Bionics Biomech.

Telemedicine has entered standard clinical practice very slowly, and the outbreak of the pandemic has led to the rapid implementation of telemedicine in most practices, which has been studied in order to better develop telemedicine technology. Through experimental research, UMPH and Blackmon found that the efficiency and durability of telehealth services depend on a variety of factors, including technology choices, government and insurance regulations, reimbursement policies, and employee and patient education and acceptance [8]. Research by May found that few centers in the adult and pediatric diabetes sector were using digital technology, telemedicine, or social media in their services [9]. To improve care and reduce costs and rapid communication between clinical staff, Ayatollahi and Ghalandarabadi used telemedicine technology to provide health care to high-risk pregnant women [10]. Jnr draws on data from the existing literature to describe the application of telemedicine and e-health as positive measures to improve clinical care [11].To make better use of telehealth technology, Eswaran and Magann described privacy concerns in telehealth issues, including barriers to care for healthcare providers and barriers for obstetric patients, licensing and payment for telehealth services, technical issues, and language barriers [12]. As telemedicine technology is unwilling to be accepted by the public, lack of forensic protocols and authoritative regulatory bodies are threatening the future of telemedicine, Nana et al. hope to establish virtual medical centers and international cooperation in the field of telemedicine and incorporate it into government programs [13]. Advanced technology has increased the use of telemedicine and information technology in disease treatment or rehabilitation, but it also requires full attention to the ethical issues in the provision of telemedicine. For this reason, Moghbeli et al. examined the ethical issues of providing telemedicine services and information technology [14]. Although many people have conducted research on telemedicine technology, few people have introduced it into the first-aid system for athletes in the marathon, which cannot make telemedicine technology be well applied. In order to solve this problem, this paper combines the two combined research.

The article "First-Aid System for Marathon Athletes Based on Telemedicine Technology" was published in 2022. Journal: Appl Bionics Biomech.

With the gradual improvement of people's material and cultural level, the marathon has become the focus of attention, and more and more people have participated in the marathon. However, since the marathon is a long-distance sport, various emergencies occur during the marathon that cause athletes to be injured. In order to provide first-aid services to the injured athletes as soon as possible, this paper provides first aid to the marathon athletes based on telemedicine technology. System was studied. While there may be barriers to using telehealth services, this type of care is feasible, and those barriers can be overcome.

## 2. Research on First-Aid System for Marathon Athletes

### 2.1. Overall frame structure of the first-aid system in the marathon

Athletes in the marathon are very prone to various situations that require treatment [15]. These situations that require treatment can be large or small, and even some situations that require treatment are not discovered and treated in the first place. It will endanger the life and health of the participating athletes. Therefore, in order to provide first aid to the injured athletes and protect the life safety of the athletes participating in the marathon, this paper studies the first-aid system in the marathon. The overall frame structure of the first-aid system in the marathon is shown in Figure 1.

As can be seen from Figure 1, the marathon field emergency system mainly consists of four parts, which mainly include workstations, data dedicated network, service terminal network, and monitoring terminal. The basic workflow of the system is that the monitoring terminal will transmit the injured athlete's information to the remote server through the dedicated data network, and the remote server will obtain the athlete's injury information and distribute the service request to each workstation through the computer network. The service information is uploaded to the server, and the server collects and processes the data and then returns it to the monitoring terminal through the data private network, thereby completing the telemedicine service and emergency service. It can be seen from the structure diagram of the first-aid system in the marathon that the private data network is the core of the whole system. On the one hand, the data private network must ensure that the correct information of athletes' injuries is transmitted to each medical workstation, and on the other hand, it must ensure that the diagnosis results and emergency medical plans are correctly transmitted to the medical staff. Each workstation is the service terminal of the entire marathon first-aid system. Their task is to obtain the injury information of athletes in time, make timely medical countermeasures, and feed back the medical information to the terminal network. The service terminal network consists of workstation hosts, firewalls, routers, and the Internet and is responsible for data fusion, processing, classification, and transmission. The monitoring terminal is mainly responsible for collecting the injury information of the athletes and transmitting the information to the data private network, so that the injured athletes can be treated in time.

The article "First-Aid System for Marathon Athletes Based on Telemedicine Technology" was published in 2022. Journal: Appl Bionics Biomech.

### 2.2. Athlete remote overall monitoring module

The athlete remote overall monitoring module generally consists of three parts [16]: the acquisition of the physiological data of the front-end subject, the transmission of the signal, and the processing of the back-end information. The front end of the module uses physiological sensors to detect the physiological information of patients, and the signals are transmitted through the Internet of Things and the Internet, and finally, the signals are processed and analyzed by the monitoring software on the host computer. The specific athlete remote overall monitoring module is shown in Figure 2.

As can be seen from Figure 2, the athlete's remote overall monitoring module is mainly composed of two parts, the marathon field monitoring network and the remote monitoring center. The athlete's physiological parameters collected by the marathon monitoring network are displayed in real time on the monitoring interface of the remote monitoring center for medical personnel to conduct analysis and research to provide necessary medical consultation services. The marathon monitoring network is mainly composed of terminal nodes, routing nodes, and community gateways. Physiological sensor nodes are various types of physiological sensors connected to the terminal nodes and routing nodes, which are installed in suitable positions of the human body to detect physiological parameter information and send the data. To the gateway of the marathon venue, the data transmission adopts the wireless communication method of the Internet of Things, which avoids the inconvenience caused by complex connections. The community gateway acts as an IoT coordinator and is located at the center of the marathon. When the venue gateway cannot directly communicate with the terminal node, the routing node forwards the communication data. The stadium gateway uploads different types of physiological data of each athlete to the network, and the remote monitoring center can access the physiological information of the players on the field through the Internet. The monitoring software of the remote monitoring center displays, stores, and analyzes the physiological parameters of the athletes in real time. When an abnormal situation occurs, the monitoring system can send an alarm signal to remind the athletes and doctors to pay attention.

The article "First-Aid System for Marathon Athletes Based on Telemedicine Technology" was published in 2022. Journal: Appl Bionics Biomech.

### 2.3. Athlete remote health monitoring module

Since the athletes in the marathon are in motion all the time [17], the traditional athlete monitoring methods cannot always pay attention to the physical and mental health of the athletes, let alone provide first-aid services for the injured athletes. In order to provide timely treatment services for injured athletes and ensure their physical and mental health, this paper studies the athlete's remote health monitoring module. The specific athlete remote health monitoring module is shown in Figure 3.

As can be seen from Figure 3, the athlete remote health monitoring module is mainly composed of three parts: a wearable multifunctional health monitoring terminal, an intelligent computer terminal, and a monitoring center service. The main function of the wearable multifunctional health monitoring terminal that athletes can carry is to monitor the athletes' ECG and blood pressure and other signals, and when necessary, the monitoring data can be sent to the central station located in the medical unit in real time. Deal with it accordingly, and receive the doctor's diagnosis and treatment advice at the same time, so that athletes can receive the same treatment and monitoring as a hospital no matter where they are. In view of the needs of system information management and simultaneous sharing and real-time monitoring by multiple users, the central station of the monitoring network is composed of a general monitoring station and an information management system. The main monitoring station is the core part of the whole system. Its main function is to receive, process, and save signals such as ECG and blood pressure from multiple injured athletes, and to real-time record, the ECG waveforms of multiple injured athletes currently connected to the monitoring center, blood pressure, and other data are displayed for reference by doctors, and at the same time, disease information can be provided to doctors, nurses, and family members of athletes for viewing. The athlete's remote health monitoring module systematically uses 5G as the information transmission carrier between the hospital monitoring center and home users. Its role is to connect the monitored patients at home and the hospital doctors, so that doctors can keep track of the patient's condition at home. There are corresponding diagnosis and treatment advice or timely rescue measures.

The article "First-Aid System for Marathon Athletes Based on Telemedicine Technology" was published in 2022. Journal: Appl Bionics Biomech.

### 2.4. Infrared pulse sensor module

Infrared pulse sensor is the latest recognition technology [18], which can be used to detect the pressure change generated by arterial pulsation and convert it into an electrical signal that can be observed and detected more intuitively. Pulse sensors are mainly used in medical equipment, teaching equipment, teaching training, and other fields, such as blood oxygen measurement, heart rate monitoring, and TCM pulse diagnosis. In order to better understand the pulse changes of athletes in the marathon field, this paper moves the infrared pulse sensor into the research of the athlete's emergency system. The specific infrared pulse sensor module is shown in Figure 3.

As can be seen from Figure 4, the infrared pulse sensor module will first control the chip to send an instruction to start the pulse signal to detect whether the athlete is injured. If the detected athlete is injured, the athlete's pulse signal will change drastically due to pain. The pulse signal that produces the drastic change is collected along with the pulse signals of other uninjured athletes. When the athletes' pulse signals are collected, they will be handed over to the signal conditioning circuit for signal conditioning. After conditioning, the conditioning circuit will connect the pulse signal to the control chip and then transmit the data to the monitoring base station after data processing. The emergency base station will process and display the received data as soon as possible. At the same time, the emergency base station will use or transmit data to the network through interfaces, so that medical staff can perform operations such as data retrieval and playback from the viewing server.

### 2.5. Athlete emergency vehicle delivery module

Since the marathon is a long-distance race, various accidents may occur during the race. These accidents may not only cause unpredictable disturbance and damage to the traditional emergency vehicle transportation route planning [19], but also delay the time for athletes to seek medical treatment in time, this paper uses the emergency vehicle transport module to study the emergency system.  Figure 5 shows the transport module of the athlete's emergency vehicle.

The article "First-Aid System for Marathon Athletes Based on Telemedicine Technology" was published in 2022. Journal: Appl Bionics Biomech.

As can be seen from Figure 5, the transport module of the athlete's emergency vehicle mainly includes three parts: the wireless local area network, the emergency vehicle, and the medical center. When an athlete is injured due to various accidents on the marathon field, the injury information will be transmitted to the computer of the medical staff on the emergency vehicle through the body sensor for the first time. After receiving the athlete's injury information, the medical staff will give information to specifically plan first-aid programs and assign existing lead vehicles and volunteer vehicles to injured athletes. During the process of transporting the injured athlete to the emergency medical center by the emergency vehicle, the medical staff on the emergency vehicle will transmit more specific injury information of the athlete to the emergency medical center through the server, so that the medical staff in the center can prepare the first-aid tools in advance and improve the first-aid efficiency. In addition, the telemedicine center will store the athlete's injury information into a database for easy recall and use.

## 3. Research on Algorithm of First-Aid System for Marathon Athletes

1. The gateway verifies the legitimacy

After adding the gateway, you need to verify the validity of its address, subnet mask, and gateway. To perform security operations on these three, you need to make sure that the previous verification passes, and then, verify the gateway. The check rule is that the address is ANDed with the subnet mask, and the network is ANDed with the subnet mask. If the result is the same, it conforms to the specification [20]. Its calculation formula is as follows:

(1) $$\begin{array}{c} e\left(P,H_{1}\left(ID\left\|PK\right.\right)\right)=e\left(g,C\right),\\ e\left(g,Y\right)=e\left(PK,{XH}_{1}{\left(ID\right)}^{\mu }\right). \end{array}$$

(2) Public key certificate processing

A public key certificate, often referred to simply as a certificate, is a digitally signed statement that binds the value of a public key to the identity of the individual, device, or service that holds the corresponding private key [21]. Its calculation formula is as follows:

(2) $$\begin{array}{c} \text{Cert}\begin{array}{c} \;\\ \text{batch} \end{array}=\prod \begin{array}{c} n\\ i=1 \end{array}\text{Cert}\begin{array}{c} \;\\ i \end{array}. \end{array}$$

(3) Define the attacker's strengths

(3) $$\begin{array}{c} \text{Adv}\left(k\right)=\left|\text{Pr}\left[b=b^{\prime }\right]-\frac{1}{2}\right|. \end{array}$$

(4) Random oracle model

Under the random oracle model, a scheme is usually designed and proven to be safe, while in the actual implementation of the scheme, a specific function needs to be used to replace the random oracle in the scheme. It should be noted that a scheme that proves security under the random oracle model is not necessarily secure in actual implementation.

(4) $$\begin{array}{c} \text{Pr}\left[B=\tilde{x}\right]=\frac{1}{\left|Z_{q}^{*}\right|}. \end{array}$$

Among them, in the case of *b* = 0 and *b* = 1, the challenge ciphertext has the same probability distribution.

(5) ECG high-pass filter

(5) $$\begin{array}{c} f_{L}=\frac{1}{2\pi *R_{12}C_{18}}. \end{array}$$

(6) Transfer function

(6) $$\begin{array}{c} A\left(s\right)=\frac{A_{0}w_{n}^{2}}{S^{2}+\left(w_{n}/Q\right)s+w_{n}^{2}}. \end{array}$$

(7) Network amplitude-frequency characteristics

(7) $$\begin{array}{c} F\left(w\right)=\frac{1-{\left(w/w_{0}\right)}^{2}}{\sqrt{{\left[1-{\left(w/w_{0}\right)}^{2}\right]}^{2}}+16{\left(1-k\right)}^{2}{\left(w/w_{0}\right)}^{2}}. \end{array}$$

(8) The transfer function of the second-order low-pass filter

(8) $$\begin{array}{c} G\left(s_{L}\right)=\frac{A_{u}{s_{L}}^{2}}{{s_{L}}^{2}+\left(1/Q\right)s_{L}+1}, \end{array}$$

where *Q* is the quality factor.

(9) Gain expression

(9) $$\begin{array}{c} A_{u}=1+\frac{R_{p}}{R_{13}}. \end{array}$$

(10) Calculation of residual energy

(10) $$\begin{array}{c} E_{r}\left(k\right)=E_{0}-\frac{\gamma t}{d_{k}+1}E_{\text{con}}. \end{array}$$

In the formula, *γ* is the comprehensive weighting factor, *d*_*k*_ is the current depth of node *k*, and *t* is the network running time.

(11) Energy consumption

(11) $$\begin{array}{c} E_{Rx}=l*E_{\text{elect}}. \end{array}$$

Among them, *E*_elect_ refers to the electronic circuit energy consumption.

(12) Packet forwarding

(12) $$\begin{array}{c} P_{A}=A+1+\left[\frac{D-A-1}{C\left(d\right)}\right]C\left(d\right), \end{array}$$

where *P*_*A*_ is the parent node address.

(13) Routing hop count

(13) $$\begin{array}{c} {RC}_{ETR}=1+d_{n}-d_{nd}+d_{d}-d_{nd}, \end{array}$$

where *d*_*nd*_is the node depth.

(14) Zero frequency gain

(14) $$\begin{array}{c} G_{0}=1+\frac{R_{f}}{R}. \end{array}$$

(15) Natural angular frequency

(15) $$\begin{array}{c} w_{n}=\sqrt{\frac{1}{R_{1}R_{2}C_{1}C_{2}}}. \end{array}$$

(16) Damping coefficient

(16) $$\begin{array}{c} \zeta =\sqrt{\frac{R_{2}}{R_{1}}}+\sqrt{\frac{R_{1}}{R_{2}}}-\left(G-1\right)\sqrt{\frac{R_{1}}{R_{2}}}. \end{array}$$

(17) Baud rate

(17) $$\begin{array}{c} \alpha =\frac{\left(256+B\_M\right)*2^{B\_E}}{2^{28}}*F, \end{array}$$

where *F* is the system clock frequency, equal to 16 MHz or 32 MHz.

(18) Gradient magnitude

(18) $$\begin{array}{c} M\left(x,y\right)=\sqrt{I\begin{array}{c} 2\\ x \end{array}+I\begin{array}{c} 2\\ y \end{array}}. \end{array}$$

(19) Gradient direction

(19) $$\begin{array}{c} \theta \left(x,y\right)=\tan^{-1}\frac{I_{y}}{I_{x}}\in \left[0,360^{{}^{\circ}}\right). \end{array}$$

The article "First-Aid System for Marathon Athletes Based on Telemedicine Technology" was published in 2022. Journal: Appl Bionics Biomech.

## 4. First-Aid Methods for Marathon Runners

### 4.1. Literature research method

Check books, periodicals, and newspapers about marathon, risk, and cognition through libraries and data platforms such as CNKI, Wanfang, and VIP browse marathon-related websites and collect, organize, read, and analyze marathon sports, risks, and cognition-related materials and policies and regulations, sort out and classify the collected data, and lay a theoretical foundation for writing this article.

### 4.2. Logical analysis method

On the basis of referring to the relevant literature, the relevant concepts are summarized and defined. Use the method of logical analysis to divide the differences and connections between concepts, syntax, and semantics, so that other related analysis can be carried out smoothly [22]. Using the combination of theory and practice, conduct research with the ideas of discovering, analyzing, and solving problems.

### 4.3. Data collection law

The data collection method is the best method used to study the emergency system, and key information can be obtained from the various emergency data collected. In order to study the first-aid system of marathon athletes more conveniently, this paper studies different first-aid systems together and compares and analyzes the performance, first-aid efficiency, and simulation parameters of these systems, so as to draw a conclusion. Corresponding data is shown in [23, 24]. In addition, for the convenience of research, this paper names the different emergency systems as system 1, system 2, system 3, system 4, and system 5, where system 5 is the system studied in this paper.

### 4.4. Data analysis method

In order to convert the various data collected into specific information related to this article, it is necessary to analyze the collected data. In order to facilitate the analysis, this paper will use a 100-point system to analyze the collected data in detail, so as to facilitate the research on the first-aid system for marathon athletes in this paper.

## 5. Experimental Research on Emergency System in Marathon

### 5.1. Research on the performance of different emergency systems

The athlete first-aid system on the marathon field is to promptly check various problems that may arise in marathon runners during long-term exercise and take corresponding measures to protect the safety of runners in emergency situations, so that runners can participate in the marathon with confidence. In order to fully guarantee the safety of athletes and provide first aid to injured athletes in the first time, the performance guarantee of the first-aid system is required. In order to study the performance of the emergency system more clearly, this paper studies different emergency systems together, and the specific data is shown in Figure 6.

The article "First-Aid System for Marathon Athletes Based on Telemedicine Technology" was published in 2022. Journal: Appl Bionics Biomech.

As can be seen from Figure 6, the performance of the emergency system is mainly composed of seven parts: transmission speed, coverage, system overhead, operating frequency, system life, network nodes, and system operation. In terms of transmission speed, system 3 and system 5 are both above 90 points, while the score of system 2 is only between 50 and 60 points, indicating that the transmission performance of system 3 and system 5 is relatively good. In terms of coverage, system 1, system 2, and system 4 are all between 55 and 68 points, indicating that the performance of this system in terms of coverage is relatively poor. In terms of system overhead, the overhead score of system 4 is the highest, at about 97 points, indicating that the overhead of system 4 is relatively large and is not suitable for long-term use. In terms of operating frequency, system life, network nodes, and system operation, the performance scores of system 3 and system 5 are much higher than those of the other three emergency systems, indicating the performance of system 3 and system 5 in these aspects is the best. On the whole, the performance of system 3 and system 5 is higher than the other three emergency systems, but the overall performance of system 3 is still lower than that of system 5, which shows that the performance of the emergency system studied in this paper is relatively good.

### 5.2. Safety analysis of different emergency systems

No matter what kind of emergency system it is, there may be various safety problems. If these potential safety problems cannot be discovered in time and solved, there may be huge safety hazards, and even athletes injured in the marathon may not receive timely treatment. In order to study the safety of the emergency system, this paper puts different emergency systems together for a comparative analysis, and the specific research data is shown in Figure 7.

As can be seen from Figure 7, the security of the emergency system mainly includes five aspects: anonymity, confidentiality, integrity, authenticity, and traceability. In terms of anonymity and traceability, the anonymity score of system 2 and system 3 is around 61 points, compared with the other three emergency systems with scores between 80 and 95, and the anonymity score of system 2 and system 3 is between 80 and 95 points. Performance and traceability are relatively low. In terms of confidentiality, the security of system 3, system 4, and system 5 is relatively high, because the scores of these three systems are all above 80 points. In terms of integrity, the security of system 1, system 4, and system 5 is higher than that of system 2 and system 3, all of which are around 90 points. In terms of authenticity, the security of system 1 and system 2 is relatively low compared to the other three emergency systems, and the authenticity of the other three emergency systems is not as good. Although the security scores of system 4 and system 5 are similar, the security score of system 4 is still lower than that of system 5 as a whole, indicating that the security of system 5 is very good.

The article "First-Aid System for Marathon Athletes Based on Telemedicine Technology" was published in 2022. Journal: Appl Bionics Biomech.

### 5.3. Emergency situations of different emergency systems for the same pain

The main purpose of the research on the first-aid system for athletes in marathons and competitions is to provide first-aid services to athletes who are injured in competitions and to protect their physical safety. In order to further study the first-aid system of athletes, this paper compares and analyzes the first-aid situation of the same pain by different first-aid systems. The specific analysis data is shown in Figure 8.

As can be seen from Figure 8, the first-aid situation is mainly composed of five parts: first-aid time, pulse measurement, system monitoring, first-aid efficiency, and first-aid route planning. Among them, for the sake of clarity, this paper adds simulated first aid to the figure and time and simulated pulse measurement data to facilitate comparative analysis. The emergency time and pulse measurement of system 1 are higher than the simulation time and measurement, indicating that the actual emergency time and pulse measurement efficiency of system 1 are relatively low, and system 1 is also relatively low in system monitoring, emergency efficiency, and route planning. The emergency time and pulse of system 2 and system 5 are slightly lower than their simulation time and measurement. These two data are roughly the same, but in terms of system monitoring, emergency efficiency, and route planning, the emergency situation of system 2 is much lower than system 5, which scores between 90 and 95 for emergency situations. The data of system 3 and system 4 in terms of emergency time and simulated emergency time, pulse measurement, and simulated pulse measurement are roughly the same as those of system 1, but differs from System 3 and System 4 in terms of system monitoring, emergency efficiency and route planning. The situation is much better than system 1. On the whole, the emergency situation of system 5 is much higher than that of the other four emergency systems, but the emergency situation of system 5 is lower than that of system 3, indicating that system 5 still has room for improvement.

The article "First-Aid System for Marathon Athletes Based on Telemedicine Technology" was published in 2022. Journal: Appl Bionics Biomech.

### 5.4. The first-aid efficiency of different first-aid systems for different injuries

The general marathon competition time is relatively long, and various emergencies are prone to occur. If these emergencies are not dealt with in time, it is easy to cause injuries to athletes, and the purpose of research on the first-aid system for marathon athletes is not just for an unexpected situation that may occur on the field; this paper studies the first-aid efficiency of different first-aid systems for different injuries, and the specific data is shown in Figure 9.

As can be seen from Figure 9, different injuries are mainly composed of seven parts: loss of consciousness, sprain, sudden trauma, fracture, dyspnea, limb injury, and collapse. In terms of loss of consciousness, the first-aid efficiency of system 2, system 4, and system 5 is better than the other two first-aid systems. In terms of sprains, the first-aid efficiency of system 1 and system 3 is about 60 points, which is far lower than the other three first-aid systems, indicating that these two first-aid systems have relatively low first-aid efficiency for sprains. In terms of sudden trauma and fracture, the first-aid efficiency of system 3 and system 5 is slightly better than that of system 4, and there is not much difference. In terms of dyspnea, the first-aid efficiency of system 1 and system 2 is inferior to the other three systems, indicating that these two systems still need to be improved before they can be used. In terms of limb injuries, the first-aid efficiency of system 3 and system are both above 90 points, indicating that the first-aid efficiency of these two systems is still relatively high, and they are valuable to a large extent. In terms of collapse state, the first-aid efficiency of system 3, system 4, and system 5 can meet the first-aid needs of athletes to a large extent. On the whole, system 2 and system 3 have different advantages and disadvantages in the first-aid efficiency for different injuries. They cannot meet the first-aid needs of athletes in the marathon at the same time. Only system 5 can meet the first-aid needs at the same time, because in system 5, the first-aid efficiency in different pain areas is above 90 points.

### 5.5. Simulation model parameter analysis of different emergency systems

The research on the first-aid system of marathon athletes based on telemedicine technology is to ensure that athletes can protect their personal safety to the greatest extent while participating in the marathon. The model parameters are studied and analyzed, and the specific unstudied data are shown in Figure 10.

The article "First-Aid System for Marathon Athletes Based on Telemedicine Technology" was published in 2022. Journal: Appl Bionics Biomech.

As can be seen from Figure 10, the simulation model parameters mainly include eight aspects: base station construction, emergency model, carrier frequency, bandwidth, subcarrier bandwidth, information collection, path loss, and control delay. System 1 has the highest parameters in emergency model and bandwidth, while the parameter values in subcarrier bandwidth, information collection, path loss, and control delay are relatively low, indicating that the simulation model parameters of system 1 are not in line with reality. First aid was needed. Although the parameters of the simulation model of system 2 are completely opposite to those of system 1, the simulation parameters of system 2 show that it is also not suitable for practical use. The simulation model parameters of system 3 are the lowest among all simulation parameter models, which shows that system 3 does not meet the needs of first aid of athletes at all. The simulation parameter models of system 4 and system 5 are roughly the same, but the parameter values of system 4 are still inferior to those of system 5, indicating that the simulation model parameter values of system 5 largely meet the needs of first aid of athletes.

## 6. Analysis of the Experimental Results of the First-Aid System for Athletes

With the gradual popularization of people's awareness of outdoor sports and physical exercise in recent years, the marathon has gradually become the focus of people's attention. However, since the competition venues of the marathon are generally from one city to another, the marathon is a sport that requires a long time and long endurance. It is precisely because of this that the athletes participating in the marathon are vulnerable to various sudden injuries caused by unexpected situations; if they are not treated in the first time, these may cause serious physical and mental damage to athletes. In order to ensure the safety of athletes, this paper studies the first-aid system for marathon athletes based on telemedicine technology.

### 6.1. Research on the Performance of Different Emergency Systems

Due to various problems and various unexpected accidents that are prone to occur in the marathon, the athletes will be injured. In order to take corresponding measures to protect the safety of the athletes in emergencies, this paper discusses the performance guarantee of the first-aid system for athletes. The results of the study suggest that systems other than the one studied in this paper have more or less disadvantages and fail to protect the health of athletes as a whole

The article "First-Aid System for Marathon Athletes Based on Telemedicine Technology" was published in 2022. Journal: Appl Bionics Biomech.

### 6.2. Safety Analysis of Different Emergency Systems

The security of the athlete emergency system mainly includes five aspects: anonymity, confidentiality, integrity, authenticity, and traceability. On the whole, different systems have a relatively low score in all aspects of safety. Only system 5 has the highest safety [25, 26] compared to the other four emergency systems, and the safety in all aspects is also relatively stable

### 6.3. The Emergency Situations of Different Emergency Systems for The Same Pain

In order to make it clearer, this paper adds two data, the simulated emergency time and the simulated pulse measurement, to the research on the emergency situation of different emergency systems for the same pain, so as to facilitate the comparative analysis. On the whole, the first-aid situation of system 5 for the same pain is much higher than the other four first-aid systems, but there is still room for improvement in system 5. Only continuous improvement and development can promote the development of the first-aid system for athletes

### 6.4. The First-Aid Efficiency of Different First-Aid Systems for Different Injuries

Compared with other data, the first-aid efficiency of system 1 for different injuries is relatively low, and the first-aid efficiency of system 3 and system 5 for different injuries is slightly better than that of system 4, and there is not much difference. On the whole, system 2 and system 3 have different advantages and disadvantages in the first-aid efficiency for different injuries. They cannot meet the first-aid needs of athletes in the marathon at the same time. Only system 5 can meet the first-aid needs at the same time, because is system 5, the first-aid efficiency in different pain areas is above 90 points

### 6.5. Analysis of Simulation Model Parameters of Different Emergency Systems

The parameters of the simulation model mainly include base station construction, emergency model, carrier frequency, bandwidth, subcarrier bandwidth, information collection, path loss, and control delay. On the whole, compared with other systems, the simulation model parameters of system 5 not only have higher scores but also are relatively stable, which can meet the first-aid needs of athletes in the marathon

## 7. Conclusion

It has been 120 years since the marathon was listed as a sports competition in the first Olympic Games. While the current marathon is in the ascendant stage of growth, it is not surprising that such or other problems have arisen. The key lies in the attitude of actively solving them. In order to provide first-aid services to injured marathon runners, this paper studies the first-aid system for marathon runners based on telemedicine technology. Through the acquisition of more image library content, images of various diseases can be extracted and learned. Finally, in the system, through image interception, the system can give corresponding diagnosis reports and store the diagnosis opinions of different diseases in the database. It can be automatically given when a diagnosis is needed, which is more intelligent, and can even help the on-site nurses to make a diagnosis without a doctor. Of course, this is only an assumption, which further supports for more hospital databases.

The article "First-Aid System for Marathon Athletes Based on Telemedicine Technology" was published in 2022. Journal: Appl Bionics Biomech.

## Figures and Tables

**Figure 1:** Overall frame structure of the first-aid system in the marathon field.

**Figure 2:** Athlete remote monitoring module diagram.

**Figure 3:** Athlete remote health monitoring module diagram.

**Figure 4:** Infrared pulse sensor module diagram.

**Figure 5:** Module diagram of athlete's emergency vehicle transportation.

**Figure 6:** Performance study of different emergency systems.

**Figure 7:** Safety analysis of different emergency systems.

**Figure 8:** The first-aid situation of different first-aid systems for the same pain.

**Figure 9:** The first-aid efficiency of different first-aid systems for different injuries.

**Figure 10:** Analysis of simulation model parameters of different emergency systems.

## Data Availability

Data sharing is not applicable to this article as no new data were created or analyzed in this study.
